# Ethnopharmacological Survey, Mineral and Chemical Content, *In Vitro* Antioxidant, and Antibacterial Activities of Aqueous and Organic Extracts of *Chamaerops humilis* L. var. argentea Andre Leaves

**DOI:** 10.1155/2022/1091247

**Published:** 2022-08-05

**Authors:** Nacima Lachkar, Fatima Lamchouri, Hamid Toufik

**Affiliations:** Laboratory of Natural Substances, Pharmacology, Environment, Modeling, Health & Quality of Life (SNAMOPEQ), Polydisciplinary Faculty of Taza (FPT), Sidi Mohamed Ben Abdellah University (USMBA) of Fez, B.P.: 1223 Taza-Gare, Taza, Morocco

## Abstract

**Introduction:**

The present study is carried out for the first time on *Chamaerops humilis* L. var. argentea Andre from the region of Taza using an ethnopharmacological survey, an experimental study of the mineralogical and chemical compositions, and evaluations of the antioxidant and antibacterial activities.

**Methods:**

After conducting the ethnopharmacological survey, a mineralogical and phytochemical study involving the preparation of aqueous and organic extracts was done. Essential oils were also extracted by hydrodistillation. Subsequently, qualitative and quantitative chemical analyses were performed. *In vitro* evaluation of antioxidant activities was performed by five tests (H_2_O_2_, DPPH, ABTS, FRAP, and RP) and antibacterial activities by the disc method and determination of MIC and MBC. A principal component analysis (PCA) was performed to visualize the different correlations.

**Results:**

The different parts of the plant are used for the treatment of digestive disorders, cardiovascular diseases, and diabetes. In addition, the leaves are rich in mineral compounds, catechic tannins, flavonoids, and sterols. However, they have some traces of essential oils. The quantitative analysis revealed that the ethanolic macerated had a higher content of total polyphenols (100.27 ± 1.95 mg EAG/g E) and catechic tannins (52.11 ± 1.02 mg EC/g E). This extract had a strong antioxidant capacity (H_2_O_2_ (37.34 ± 0.55%), DPPH (IC_50_ = 31.18 ± 0.66 *μ*g/ml), ABTS (108.28 ± 1.29 mg E AA/g E), FRAP (148.85 ± 0.43 mg E T/g E), and RP (10.86 ± 0.01 mg E AA/g E). The same extract had a bactericidal effect against *Staphylococcus aureus*. Principal component analysis (PCA) showed that antioxidant activity was highly correlated with the chemical composition of *C. humilis* leaves; a high correlation was recorded between the total polyphenol content and ABTS (*r* = 0.9779), FRAP (*r* = 0.9644), DPPH (*r* = 0.9418), and PR (*r* = 0.9271) tests. In addition, cathectic tannins were highly correlated with the tests of DPPH (*r* = 0.9753) and ABTS (*r* = 0.8843). Flavonoids were similarly correlated with DPPH (*r* = 0.8897) and ABTS (*r* = 0.7599) tests.

**Conclusion:**

These results could justify the traditional use of the leaves of *Chamaerops humilis* in the region of Taza for the treatment of some diseases.

## 1. Introduction

For several years, the use of herbal preparations has been of great importance in the therapeutic field. We also notice that this sector concerns the developed countries as well as the developing countries. For the first countries, the mistrust towards synthetic products and the desire to consume organic extracts are the main factors that encourage them to use medicinal and aromatic plants in their daily life. In the United States of America, for example, 25% of prescribed medicines are plant based [1]. In Europe, the number of food supplements produced from plants has grown exponentially in 2002 [2]. Developing countries consider traditional medicine as part of the cultural heritage; the population of these countries has a know-how related to the uses of plants in traditional pharmacopoeia. Similarly, they use medicinal plants and herbal remedies for economic reasons related to purchasing power which is low, difficulties in accessing health care due to the high cost of synthetic drugs.

In Morocco, ensuring access to primary health care and universal health coverage for the population remains a major challenge. Despite the efforts made in recent years, the problem of access to health care is far from being solved, which pushes the population to seek other accessible and less expensive means for the treatment of diseases, including medicinal plants. Indeed, Morocco has a very important floristic wealth characterized by a great diversity of plants with 4200 species and a large number of species and subspecies [3]. This natural wealth places Morocco in an important position among other Mediterranean countries. Morocco also has a long history in phytotherapy especially in rural areas [4].

Similarly, the region of Taza (north-east Morocco) has an important natural richness and a local traditional know-how related to the uses of medicinal plants in phytotherapy [5, 6]. *Chamaerops humilis* L. var. argentea Andre is among the very abundant plants in the region of Taza and is the only palm species naturally distributed in Europe and Africa [7]. In Europe, *Chamaerops humilis* is present on the coasts of southern Portugal, southern and eastern Spain, south-eastern France, and western Italy [8, 9]. The species is also found on most of the large islands in the western Mediterranean, namely, the Balearic Islands, Sardinia, Sicily, and Malta. In Corsica, it does not seem to be indigenous [10]. In Africa, it is mainly located in Morocco but also in northern Algeria and northern Tunisia. The species has the widest distribution in Morocco, where 2 varieties have been distinguished: a green-leaf form (var. *humilis*) and a glaucous-leaf form (var. argentea André) [9, 11, 12]. First, *C. humilis* or dwarf palm belongs to the Arecaceae family (Palmaceae), it is small in size and can grow up to 1.5 m, it is a dioecious plant, its leaves are palmate and sclerophyllous [13], and the fruits are “polydrupes” that ripen in autumn (September–November). They are attached to inflorescences up to 30 cm long (37–91 fruits per branch), and the female inflorescences are solid, brownish, and bear fruits or only the calyx; in contrast, the males have smaller and very fragile inflorescences [14].

In addition to the abundance of the variety *Chamaerops humilis* L. var. argentea Andre in the region of Taza. To our knowledge, no ethnopharmacological survey nor mineralogical analysis or studies of the chemical composition and antibacterial activity have been carried out on *Chamaerops humilis* L. var. argentea Andre in the region of Taza. In Morocco, we identified from the literature only one preliminary study made on the species *Chamaerops humilis* on a single extract and only one test of antioxidant activity [15]. In Algeria, an ethnopharmacological study was conducted on the species *Chamaerops humilis* [16] and another on the chemical composition of the species *Chamaerops humilis* [17], and finally, another ethnobotanical study was conducted still in Algeria on *Chamaerops humilis* variety argentea André but without going to pharmacological tests to assess the traditional uses mentioned by the respondents [18]. Studies have declared the use of the plant in phytotherapy; the aerial part is against pyelonephritis and prostatitis [19]; the fruits and roots are also used to treat type 2 diabetes [20], the plant is also used for the treatment of digestive system disorders and in veterinary medicine [21]; the fruits are used as antidiarrheal medicine [22] and to treat digestive system disorders in general [23]. Digestive disorders are typically associated with a long line of acute and chronic human diseases [24]. The digestive system contains intestinal microbiota that includes all the bacteria that live in symbiosis and have a crucial role in the digestion of food. Any imbalance can lead to an increase in the proliferation of pathogenic bacteria, and consequently, a change in the composition of the microbiota of the gastrointestinal tract can lead to hypochlorhydria [25], to abdominal discomfort, bloating, and diarrhea, which can cause hypophosphatemia and hypomagnesemia that affect the normal functioning of our organs [26–28]. In addition, researches have reported the role of minerals for the proper functioning of the digestive system; the increase of dietary calcium reduces the risk of developing colon adenomas, a reduction in the risk of colorectal cancer [29]. In addition, the various fermentation processes in the rumen require an adequate supply of minerals [30].

Faced with this observation and these data, we were interested in conducting a global study on *Chamaerops humilis* L. var. argentea Andre to highlight its therapeutic interest by adopting the ethnopharmacological approach. Thus, we were interested on the one hand in the study of the interest of *C. humilis* in traditional medicine via an ethnopharmacological survey conducted in the province of Taza and, on the other hand, to carry out an analysis of its mineralogical and chemical composition and a study of biological activities in order to confirm or deny the use of this plant in traditional medicine. The chemical study included aqueous extraction (decoction, infusion, and maceration) and organic extraction with Soxhlet and cold by three solvents (ethanol, chloroform, and hexane), the screening of secondary metabolites, and the quantification of phenolic compounds.

The biological study consisted of an *in vitro* evaluation of the antioxidant activity by five tests: hydrogen peroxide scavenging test (H_2_O_2_), DPPH (2,2-diphenyl-1-picrylhydrazil) free radical scavenging test, ABTS (2,2-azinobis (3-ethyl-benzothiazoline-6-sulphonate) or TEAC (Trolox equivalent antioxidant capacity), ferric-reducing antioxidant power assay (FRAP), and the reducing power (RP) test. And then, a study on antibacterial activity by the disc method and the determination of minimum inhibitory concentrations (MIC) and minimum bactericidal concentrations (MBC) was done. Finally, a principal component analysis (PCA) was performed to investigate the correlations between the chemical composition of the different extracts and their biological activities and also between the five tests used for the evaluation of the antioxidant activity.

## 2. Material and Methods

### 2.1. Ethnopharmacological Survey

#### 2.1.1. Study Site

The province of Taza is located in northeastern Morocco east of the Fez-Meknes region, situated between the Pre-rif in the north and the Middle Atlas in the south, characterized by a semicontinental climate with a Mediterranean influence [31].

The province is characterized by a remarkable diversity and natural wealth because it has one of the oldest national parks in Morocco: the Tazekka National Park [32].

#### 2.1.2. Data Collection

The ethnopharmacological survey was conducted in four stations in the province of Taza: Taza city, Bab El Mrouj, Gueldaman, and Bab Boudir. The choice of survey stations was based on their abundance of *Chamaerops humilis* L. var. argentea Andre that makes its traditional use easy and therefore allows the accumulation of traditional knowledge by the local population (Figures 1 and 2).

The method used was a questionnaire developed and adopted by the Laboratory of Natural Substances, Pharmacology, Environment, Modeling, Health and Quality of Life (SNAMOPEQ), Polydisciplinary Faculty of Taza, Sidi Mohamed Ben Abdellah University (USMBA) of Fez, Morocco [5, 6, 33]. The survey was conducted using a questionnaire with a simple choice, multiple choice, and open-ended questions about the informant and *C. humilis* and its medicinal aspects. The questions were written in French language, and due to the fact that the province of Taza is with multiple tribes (Branès, Ghiata, Tsoul, and the Amazighs) and each tribe is individualized by a separate dialect and to avoid difficulties in understanding the questions, we helped the informants to understand the questionnaire with their own dialects (Arabic/Amazigh) [33–38]. The data obtained were later translated into French and English [39]. The survey was conducted among traditional practitioners, herbalists, farmers, nomads, and a total of 239 people.

The information collected concerned the profile of the respondent (age, gender, and level of education) and ethnopharmacological data such as the vernacular name of the plant, part used, methods of preparation, and uses of the plant.

### 2.2. Mineralogical and Chemical Compositions

#### 2.2.1. Plant Material

The plant material consists of the leaves of the plant *Chamaerops humilis* L. var. argentea Andre collected in February 2017 from the mountains of Bab Boudir at 42.3 km from the city of Taza, geographical coordinates N 34°405.635′, W 004°05.900′, altitude: 1358 meters (Figure 1).

The botanical identification of the plant *Chamaerops humilis* L. var. argentea Andre was made by Dr. Abdelmajid Khabbach, botanist at the Laboratory of Natural Substances, Pharmacology, Environment, Modeling, Health and Quality of Life (SNAMOPEQ), at the Polydisciplinary Faculty of Taza, based on the works of Valdés and his collaborators and Richard [40, 41] (Figure 3).

A reference sample SB2017 of the leaves of *Chamaerops humilis* L. var. argentea Andre was deposited in the herbarium of the SNAMOPEQ of the Polydisciplinary Faculty of Taza, Morocco.

#### 2.2.2. Mineralogical Study

The quantitative analysis of mineral elements was done according to the protocol of Arora and collaborators [42]. The test procedure has been described in detail in our previous work [43–45].

### 2.3. Phytochemical Study

#### 2.3.1. Preparation of Extracts

The extraction of bioactive molecules contained in the leaves of *C. humilis* was carried out by two methods: an aqueous extraction with distilled water in three ways: decoction, infusion, and maceration, and another organic one by hot Soxhlet using organic solvents of different polarities (ethanol, chloroform, and hexane) and cold by maceration in ethanol. The extraction procedure employed is detailed in our previous work [43].

After removing the solvents under reduced pressure at 40°C in a Buchi R-210 Rotavapor, all extracts obtained were weighed for yield calculation and stored at 4°C until use.

#### 2.3.2. Extraction of Essential Oils by Hydrodistillation

The extraction of essential oils was performed by hydrodistillation using the Clevenger apparatus. The leaves of *Chamaerops humilis* var. argentea André are immersed in a flask containing distilled water, and then, the whole is brought to boil using a flask heater.

#### 2.3.3. Phytochemical Screening

Phytochemicals were characterized on both the powdered plant material and the aqueous and organic extracts of the plant using staining and precipitation reactions as described by a previous work in our laboratory [43, 44, 46–49]. The characterization reagents were used to investigate the following chemical groups: catechic tannins and gall tannins using the ferric chloride FeCl_3_ reaction [50], flavonoids using the cyanidine reaction [51], saponins using the foaming technique [52], alkaloids by two reagents, Dragendorff (potassium iodobismuthate) and Valser-Mayer (potassium tetraiodomercurate) [53], sterols with the Liebermann reaction [51], anthracenosides by the Borntraeger reaction [54], free quinones by sodium hydroxide [55], and anthraquinones with potassium hydroxide for plant material and with ammonia solution for aqueous and organic plant extracts [56].

#### 2.3.4. Quantification of Phenolic Compounds

The results of phytochemical screening of *C. humilis* leaves directed us in the quantification of total polyphenols, flavonoids, and catechic tannins according to the protocols described in previous works of our laboratory [43, 44, 46–49].

*(1) Determination of Total Polyphenols*. The determination of total polyphenols in the extracts of *C. humilis* leaves was performed according to the Folin-Ciocalteu reagent method [57]; the test protocol is described in previous publications [43, 47, 49, 58]. The total polyphenol content of the extracts was expressed as microgram (*μ*g) equivalent of gallic acid per milligram (mg) of extract (*μ*g GAE/mg E).

*(2) Determination of Flavonoids*. Total flavonoids were quantified using the technique adapted by Mihai and collaborators with aluminum trichloride and soda [59]; the methodology for the quantification of flavonoids is detailed in previous works [49, 57]. The flavonoid content was expressed as *μ*g quercetin equivalent/mg extract (*μ*g QE/mg E).

*(3) Determination of Catechic Tannins*. Catechin tannins are determined by the vanillin method using the procedure reported by Joslyn [60]. This method is based on the ability of vanillin to react with condensed tannin units in the presence of acid to produce a colored complex measurable at 500 nm. The detailed protocol is described in our previous work [35, 46–48]. Tannin concentration was expressed as microgram equivalents of catechin per milligram of extract (*μ*g CE/mg) from the calibration curve.

#### 2.3.5. Antioxidant Activity

The determination of the antioxidant capacity of aqueous and organic extracts of the leaves of *C. humilis* was carried out *in vitro* by five tests: hydrogen peroxide scavenging test H_2_O_2_, free radical scavenging test DPPH (2,2-diphenyl-1-picrylhydrazil), ABTS (2,2-azinobis (3-ethyl-benzothiazoline-6-sulphonate) method or TEAC (Trolox Equivalent Antioxidant Capacity), iron reduction antioxidant capacity (FRAP), and the reducing power test (PR).

*(1) Hydrogen Peroxide Scavenging Assay (H_2_O_2_)*. The study of H_2_O_2_ scavenging activity was performed by the method described by Ruch and collaborators [61]; the experimental protocol was described by later works [43, 44, 46–49]. The results are expressed as percent inhibition according to the following formula:

(1) $$\begin{array}{c} \%{\text{H}}_{2}{\text{O}}_{2}\text{ scavenging}=\left[\frac{\left(\text{AC}-\text{AT}\right)}{\text{AC}}\right]\times 100\left[6\right], \end{array}$$

where *AC* is the absorbance of the control and AT is the absorbance of the test.

*(2) Determination of the Antifree Radical Activity by the DPPH Test*. The activity of the DPPH radical scavenging (2,2-diphenyl-1-picrylhydrazyl (C_18_H_12_N_5_O_6_) from the nine aqueous and organic extracts of *C. humilis* is determined according to the method of [62], described by previous studies from our laboratory [43, 44, 46–49]. The results obtained were compared to the DPPH scavenging activity for Trolox, BHT, and ascorbic acid which were used as reference standards. The results are expressed as percent inhibition using the following formula:

(2) $$\begin{array}{c} I\left(\%\right)=\left[\frac{\left(\text{Abs}-\text{Abse}\right)}{\text{Abs}}\right]\times 100, \end{array}$$

where *I* (%) is the percent inhibition, Abs is the absorbance of negative control, and Abse is the absorbance of the sample.

The IC_50_ (50% inhibitory concentration) is the concentration of the tested sample capable of reducing 50% of the DPPH^−^ radical which was determined graphically from the percentage of scavenging effect versus the corresponding sample concentration.

*(3) Trolox Equivalent Antioxidant Capacity Using ABTS (TEAC)*. The evaluation of the ABTS^−^ radical scavenging capacity was determined by the method of [63]. The technique of this assay has been detailed in our subsequent work [43, 44, 46–49]. The total antioxidant capacity of the 9 aqueous and organic extracts of the plant was expressed as mg of Trolox equivalent per gram of extract (*μ*g of TE/mg E).

*(4) Ferric-Reducing Antioxidant Power Assay (FRAP)*. Determination of the iron reduction antioxidant capacity (FRAP) of our 9 aqueous and organic extracts was determined according to the method described by Benzie and Strain [64]. The detailed protocol refers to several references from our previous studies [43, 44, 46–49]. Results are expressed as micrograms of Trolox equivalent per milligram of extract (*μ*g TE/mg E).

*(5) Reducing Power Assay (RP)*. The reducing power of iron was determined according to the method of Oyaizu [65]. The experimental protocol was detailed in our previous work [43, 44, 46–49]. Results are expressed as *μ*g ascorbic acid equivalent per milligram of extract (*μ*g EAA/mg E).

#### 2.3.6. Antibacterial Activity

The antibacterial activity evaluation tests were performed on *Staphylococcus aureus* CECT976, *Bacillus subtilis* DSM6633, and *Listeria innocua* CECT 4030 for Gram^+^ bacteria and *Escherichia coli* K12, *Proteus mirabilis*, and *Pseudomonas aeruginosa* CECT118 for Gram^−^ bacteria. The evaluation of the antibacterial activity of the different organic extracts was carried out by two methods, the disc diffusion method in an agar medium, and then the determination of the minimum inhibitory concentration (MIC) and the minimum bactericidal concentration (MBC).

*(1) Agar Diffusion Method*. Organic extracts at concentrations of 40, 80, and 100 mg/ml were prepared and dissolved in 10% dimethyl sulfoxide (DMSO).

Microbial suspensions in the exponential phase of growth (approximately 10^8^ CFU/m according to the McFarland scale) were plated on sterile Mueller Hinton agar contained in the petri dishes. Sterile Whatman paper discs with a diameter of 6 mm impregnated with 40 mg/ml, 80 mg/ml, and 100 mg/ml of organic extracts were aseptically deposited on the seeded agar, and then, the plates were incubated at 37°C for 24 h. Antibacterial activity is determined by measuring the diameter of the inhibition zone around each disc. The experiment was performed in triplicate for each microbial species. 10% DMSO was used as a negative control, and tetracycline and Amikacin were used as positive controls [66].

*(2) Macrodilution Method in Liquid Medium*. *(2)1. Determination of the Minimum Inhibitory Concentration (MIC)*. The MIC is the lowest concentration of a substance that can inhibit the growth of bacteria for 18 to 24 hours at 37°C. The MIC was performed only for extracts that have shown sensitivity during the agar diffusion method. It was evaluated by the microdilution method in agar medium. The initial concentration was 80 mg/ml.

100 *μ*l of liquid culture medium (Mueller-Hinton) was introduced in each well, then, 100 *μ*l of the extracts to be tested was added, and successive dilutions were carried out. Finally, the wells were inoculated with 10 *μ*l of the suspension of microorganisms at final inoculum concentrations of 10^8^ CFU/ml.

The microplate was covered and incubated at 37°C for 24 hours. 10 *μ*l of MTT (3-(4,5-dimethylthiazol-2-yl)-2,5-diphenyl tetrazolium bromide) solution was added to each well; after a 15 minute reincubation at 37°C, the reading was taken. The appearance of a purple coloration shows bacterial growth. The MIC is the lowest concentration of the test substance at which no visual disturbance is observed [67].

*(2)2. Determination of the Minimum Bactericidal Concentration (MBC)*. In order to determine the MBC values, we used well solutions with an extract concentration equal to or higher than the obtained MIC values. 10 *μ*l of each well was plated on Mueller-Hinton medium in petri dishes. After incubation for 24 to 37°C, the MBC, defined as the lowest concentration showing no bacterial growth, was determined.

#### 2.3.7. Data Analysis

For the ethnopharmacological survey, the data recorded on the forms used for the survey were then processed and entered into the Excel software. The analysis of the data used descriptive statistics methods. Thus, the qualitative variables are described using the numbers and percentages by the following formula:

(3) $$\begin{array}{c} \text{Frequency in}\%=\left(\frac{\text{xi}}{N}\right)*100, \end{array}$$

where xi is the number of employees of a given value and *N* is the total number of employees.

The statistical analysis of the data was done using the one-way analysis of variance (ANOVA) followed by the Tukey post test. All the results obtained were expressed as mean ± standard deviation. All results were analyzed using GraphPad Prism 5 statistical analysis software, and differences were considered statistically significant for *p* < 0.05 in all statistical analyses.

Principal component analysis (PCA), developed by Pearson, was also used to analyze the correlations between the chemical composition of the aqueous and organic extracts prepared from the leaves of *C. humilis* and their biological activity and also between the different tests used for the evaluation of the antioxidant activity.

## 3. Results

### 3.1. Ethnopharmacological Study

#### 3.1.1. Information about the Respondents

The analysis of the information collected on the respondents made it possible to obtain data on age, gender, and level of education.

*(1) Age Factor*. According to the data analysis, the average age of the respondents is 50 years. The frequency of use of *Chamaerops humilis* L. in traditional medicine changes with the age group, and people over 70 years old has the highest frequency of use with a percentage of 100%. Followed by the age groups [50-69 years] and [30-49 years] with frequencies of 90.74 and 81.19% respectively (Figure 4).

*(2) Gender Factor*. The survey was conducted among 239 people who are divided into 144 men and 95 women. The results obtained show that they have a frequency of users of *C. humilis* very close, and it is 84.21% for women and 90.27% for men (Figure 5).

*(3) Level of Study*. The data obtained show that there is a significant effect on the level of education of the populations surveyed on the frequency of medicinal use of *C. humilis*; the vast majority of users of *C. humilis* are illiterate with an average of 65.27% (Figure 3). This category presents a percentage of 89.10% regarding the traditional therapeutic use of the studied species. However, people with primary and secondary education have a significant percentage of use which is 88.57% and 55.55%, respectively, while those with university education use this medicinal plant very seldom with a percentage of 25% (Figure 6).

#### 3.1.2. Vernacular Names of *C. humilis*

According to the population surveyed, in the Arabic dialect, the entire plant is known by the name Doum or “Douma” to designate a single plant or “Tigztamet” in Amazigh. Each part of the plant also has a distinct vernacular name; the leaves are called “Dûm” or “Laâzaf” in Arabic dialect, and the fruits are called “Lghaz” and “Ghaz dûm” in Arabic dialect or “Aghaz” in Amazigh. The palm heart is called “Jammar” or “Jammara” to refer to a single unit of the palm heart in dialectal Arabic; in Amazigh, it is called “Agnit” and the spadix is called “Al baâouche” in dialectal Arabic or “Timjjat wgnit” or “Timjjin wgnit” as a single spadix in Amazigh.

#### 3.1.3. Medicinal Interest of *C. humilis*

The medicinal interest of *C. humilis* concerned several aspects such as the part used, the disease treated, the mode of preparation, and other uses of this plant in the Moroccan traditional medicine.

*(1) Parts Used of C. humilis*. The results obtained (Figure 4) show that heart of palm and spadice are the most used parts in the four surveyed stations with a similar percentage of 79.49%, followed by fruits, leaves, and roots with percentages of 24.26%, 8.78%, and 4.60%, respectively. In addition, during the survey, we noticed that most of the respondents do not differentiate between the two parts, heart of palm and spadice; they usually mention of the heart of palm, except in the last station of «Bab Boudir» (Figure 7).

*(2) Diseases Treated by C. humilis*. The analysis of the information collected by the surveys carried out in the four survey stations shows that the three parts, palm heart, spadice, and fruits, are used for the treatment of digestive disorders (bloating, ulcer, intestinal worms, and inflammations), diabetes, cardiovascular system disorders, respiratory system disorders, and hepatitis. In addition, the fruits are also used to solve fertility problems, especially in women, and to strengthen the immune system. The roots are used for the treatment of digestive disorders and diabetes and in association with *Lawsonia inermis* or “natural henna” (belonging to the family Lythraceae, genus *Lawsonia*, species *inermis*) against hair loss. Our data indicate that the leaves are also used to treat digestive system disorders in humans and livestock (Table 1).

*(3) Preparation Method of C. humilis*. During the survey, we found that palm heart and spadice are generally used raw without preparation with a percentage of 95.38% and can be used roasted, in decoction or in combination, with a percentage of 2.56%, 1.02%, and 1.02% (Figure 8).

The fruits are also used raw with a percentage of 59.32% or in association with pure honey or olive oil (38.98%); they are weakly used in decoction (1.69%). On the other hand, we found that the decoction dominates as a method of preparation of the roots (90.90%) and the infusion of the roots is less used with a percentage of 9.09%.

The leaves are crushed and used with a percentage of 47.82%, in decoction with 34.78% and in aqueous maceration with 17.39%.

*(4) Other Uses of the Plant C. humilis*. The data obtained from the surveys carried out in the four stations show that saw palmetto has several uses other than medicinal. This species can serve as food for humans (palm heart, spadice, and fruit) and food for animals (leaf and fruit); the leaves are used extensively for the manufacture of handicrafts and can be used as a tool for washing dishes (a type of sponge). Also, they are used in the past for the production of vegetable hair, the leaves and fruits are also used to practice magic, and the whole plant is used as firewood (Table 2).

### 3.2. Mineralogical Analysis of *Chamaerops humilis* L. var. argentea Leaves

Mineralogical analysis by inductively coupled plasma atomic emission spectrometry (ICP-AES) revealed the presence of iron, potassium, phosphorus, magnesium, sodium, copper, calcium, zinc, selenium, and strontium (Table 3).

Table 3 illustrates the results of the study of mineral contents of the leaves of *C. humilis*. The analysis of minerals showed that this plant contains significant contents of iron, potassium, phosphorus, and magnesium with values of 82395.00, 9354.9, 1828.62, and 1312.47 mg·kg^−1^, respectively. Sodium, copper, calcium, and zinc are present in average amounts with values of 627.03, 542.64, 92.19, and 66.15 mg·kg^−1^, respectively. Selenium and strontium are present with low levels of about 3.00 mg·kg^−1^ for each.

### 3.3. Phytochemical Study

#### 3.3.1. Yields of Aqueous and Organic Extractions

Aqueous and organic extraction of *C. humilis* leaves resulted in the yields presented in Table 4.

From the results in Table 4, we can observe that organic extraction gives the slightly better yields compared to aqueous extraction and that hot extraction gives the best yields compared to cold extraction by maceration for both aqueous and organic extraction modalities.

For aqueous extracts, the decocted (10%) is richer in extractable matter followed by the infused (2.2%) and the macerated (1.2%). For organic extracts, the best yield was obtained by the most polar solvent and ethanol hot by Soxhlet (10.84%), followed by ethanolic macerated (3.18%), then chloroformic extract (1.245%), followed by chloroformic macerate (1.040%) and hexanic extract (0.820%), and lastly hexanic macerate (0.433%).

#### 3.3.2. Extraction by Hydrodistillation

The extraction by hydrodistillation of essential oils from the leaves of *Chamaerops humilis* var. argentea André gave only a few traces that are stuck to the internal surface of Clevenger. The extraction yield was not determined due to the small amount extracted.

#### 3.3.3. Phytochemical Screening

Phytochemical screening was carried out on the powder and on the aqueous and organic extracts of the leaves of *C. humilis*. The tests carried out are aimed at highlighting the presence of chemical families: catechic tannins and gall tannins, flavonoids, saponins, alkaloids, sterols, anthracenosides, free quinones, and anthraquinones, and the results obtained are represented in Table 5.

The results of phytochemical screening carried out on the powder of plant material and different aqueous and organic extracts of the leaves of *C. humilis* are mentioned in Table 5. The powder of the leaves of *C. humilis* contains the catechic tannins, flavonoids, saponins, sterols, and free quinones. Concerning the aqueous extracts, the decocted and infused contain catechic tannins, flavonoids, and saponins and the decocted contains in addition the free quinones, whereas the macerated, cold-prepared extract contains only the catechic tannins and saponins.

For the organic extracts, ethanolic extract and ethanolic macerated contain catechic tannins, flavonoids, saponins, and free quinones; chloroformic extract and chloroformic macerate contain catechic tannins; hexanic extract and hexanic macerate contain catechic tannins and sterols. For the other families of secondary metabolites, gall tannins, alkaloids, anthracenosides, and anthraquinones are absent in both the leaf powder and in all the aqueous and organic extracts prepared from them (Table 5).

#### 3.3.4. Phytochemical Dosage

The secondary metabolites to be assayed (total polyphenols, flavonoids, and catechic tannins) were selected based on the results of phytochemical screening of leaves of *C. humilis*. The results of the assay are presented in Table 6.

The results of quantitative analyses of phenolic compounds in aqueous and organic extracts of *C. humilis* leaves are reported in Table 6. The organic extracts contain high contents of total polyphenols, flavonoids, and catechic tannins compared to the aqueous extracts. For the aqueous extracts, the decocted has the highest content of total polyphenols of 13.23 ± 0.19 mg EAG/g E in comparison with the infused (2.11 ± 0.03) and macerated (2.02 ± 0.04) with a statistically significant difference.

For the organic extracts, we found that the total polyphenol contents of the different organic extracts varied between 20.8 ± 1.33 and 100.27 ± 0.66 mg EAG/g E. The highest concentration of phenols was measured in the ethanolic macerated, with a level of 100.27 ± 1.95 mg EAG/g E and the hot Soxhlet-prepared ethanolic extract (96.99 ± 0.82 mg EAG/g E) with a statistically insignificant difference, followed by the chloroformic and hexanic macerates, respectively, with a statistically insignificant difference and lastly the chloroformic and hot prepared hexanic extracts, with values of: 37.51 ± 1.66, 34.77 ± 1.19, 28.04 ± 0.43, and 20.8 ± 1.33 mg EAG/g E with a statistically significant difference.

#### 3.3.5. Determination of Flavonoids

Concerning the aqueous extracts, we found that the decocted has the highest flavonoid content (56.36 ± 0.39 mg EQ/g E), followed by the infused (41.94 ± 0.09 mg EQ/g E) and lastly the aqueous macerate (4.48 ± 0.26 mg EQ/g E) with a statistically nonsignificant difference between the three extracts. For the organic extracts, the chloroformic macerate has high flavonoid contents with 542.7 ± 24.03 mg EQ/g E, followed by the ethanolic macerated (468.25 ± 9.07 mg EQ/g E) and the ethanolic extract (457.98 ± 5.18 mg EQ/g E) prepared by hot Soxhlet with a statistically significant difference. The chloroformic extract and the hexanic macerate present flavonoid contents of 356.87 ± 10.90 and 335.48 ± 10.67 mg EQ/g E, respectively, with a statistically nonsignificant difference and lastly the hexanic extract with a content of 273.25 ± 8.92 mg EQ/g E (Table 6).

#### 3.3.6. Determination of Tannins

The results presented in Table 6 reveal that the decocted has a significant amount of catechic tannins (10.08 ± 0.07), followed by the infused (1.28 ± 0.03) and lastly the macerated (1.26 ± 0.04) with a statistically nonsignificant difference between the three aqueous extracts. For organic extracts, ethanolic macerated is highly rich in tannins with a value of 52.11 ± 0.24 mg EC/g E, with a statistically nonsignificant difference with ethanolic extract (50.27 ± 0.99 mg EC/g E), followed by chloroformic macerate, chloroformic extract with a nonsignificant difference, and lastly hexanic macerate and hexanic extract with a nonsignificant difference, with values of 39.05 ± 0.78, 35.72 ± 2.35, 30.16 ± 1.02, and 25.5 ± 0.51 mg EC/g E (Table 6), respectively.

#### 3.3.7. Antioxidant Activity

Antioxidant activity was evaluated for aqueous and organic extracts of *C. humilis* leaves using H_2_O_2_, DPPH, ABTS, FRAP, and RP assays. The results obtained are presented in Table 7.

*(1) Hydrogen Peroxide Scavenging Assay (H_2_O_2_)*. The results obtained revealed that all the extracts have a strong capacity to neutralize hydrogen peroxide clearly superior to the reference drug ascorbic acid (14.35 ± 0.002%) at a concentration of 100 *μ*g/ml and the decocted (aqueous extract) proved to be the most active (45.77 ± 0.15%) compared to all the extracts tested and its activity is three times higher than that of ascorbic acid.

For aqueous extracts, in comparison with decocted (45.77 ± 0.15%), the infused came second (29.65 ± 0.31%) with statistically significant difference, followed by aqueous macerate (29.24 ± 0.62%) with statistically insignificant difference with the infused and significant with the decocted. The decocted presented a high hydrogen peroxide inhibition value compared to those of the organic extracts with a statistically significant difference. Regarding the organic extracts, ethanolic macerated showed a high hydrogen peroxide inhibition rate followed by hot methanolic extract with statistically insignificant difference, followed by chloroformic macerate and chloroformic extract with statistically insignificant difference; hexanic extract shows statistically insignificant difference with chloroformic macerate with inhibition percentages of 37.34 ± 0.55, 36.80 ± 0.33, 35.79 ± 0.29, 34.83 ± 0.26, and 33.96 ± 0.17%; the hexanic macerate comes last with 21.59 ± 1.14% and with a statistically significant difference with all the tested extracts (Table7).

*(2) 2,2-Diphenyl-1-Picrylhydrazil Free Radical Scavenging Activity (DPPH)*. The lowest IC_50_ value corresponds to the highest extract efficiency. The DPPH free radical scavenging capacity is proportional to the increase in concentration of the tested samples. Both aqueous and organic extracts of *C. humilis* leaves show significant capacity to scavenge the DPPH free radical (Table7). For the aqueous extracts, the decocted shows the highest capacity to scavenge the free radical with an IC_50_ value of 6814 ± 0.08 *μ*g/ml, followed by the macerate (9260 ± 0.39 *μ*g/ml) and then the infused (10280 ± 0.04 *μ*g/ml) with a statistically significant difference between the three extracts. The organic extracts have a significantly higher free radical capacity than the aqueous extracts with a statistically significant difference. Ethanolic macerated exhibited the best activity with an IC_50_ of 31.18 *μ*g/ml ± 0.66 followed by hot ethanolic extract, hexanic macerate, hot chloroformic extract, chloroformic macerate with a statistically insignificant difference, and lastly hot hexanic extract which exhibits a statistically significant difference with the other organic extracts and the IC_50_ are 44.25 ± 2.31, 335.1 ± 0.5, 490.06 ± 0.54, 491.53 ± 2.08, and 975.83 ± 11.83 *μ*g/ml).

From these results, it seems that via the DPPH test, all the extracts studied have an antioxidant activity but lower than that of the reference standards (BHT, Trolox, and ascorbic acid) with a statistically significant difference (Table 7).

*(3) ABTS^+^ Radical Scavenging Test*. Aqueous extracts recorded a low antiradical potency towards the ABTS radical; decocted comes first with a value of 14.44 ± 0.003 mg TE/g E, followed by infused (2.49 ± 0.19 mg TE/g E) and aqueous macerated (2.46 ± 0.05 mg TE/g E) with a statistically nonsignificant difference between the three extracts. For the organic extracts studied, the best antiradical activity is recorded for ethanolic macerated (108.28 ± 1.29 mg TE/g E) and ethanolic extract (78.21 ± 0.98 mg TE/g E) with a statistically nonsignificant difference; chloroformic extract and chloroformic macerate present a scavenging activity of the ABTS^+^ radical of 30.1 ± 0.75 and 41.93 ± 0.62 mg TE/g E, respectively, with a statistically significant difference. Hexanic extract and hexanic macerate showed considerable antiradical capacities of 14.87 ± 2.31 and 30.15 ± 3.76 mg TE/g E, respectively, with a statistically significant difference (Table 7).

*(4) Ferric-Reducing Antioxidant Power Assay (FRAP)*. The antioxidant activity of an extract by the FRAP method corresponds to the capacity of this extract to reduce Fe^3+^ to ferrous ion (Fe^2+^), which is reflected by the increase in absorbance at 593 nm. The results obtained show that the iron reduction capacity varies according to the extracts; for the aqueous extracts, the decocted has a reducing activity of 23.44 ± 0.07 mg TE/g E, followed by the infused (6.67 ± 0.017 mg TE/g E) and lastly the macerated (5.34 ± 0.14 mg TE/g E); the aqueous extracts present a statistically significant difference. In addition, the decocted showed a high capacity of reduction of ferric ions (Fe^3+^) in comparison with three organic extracts: chloroformic extract, chloroformic macerate, and hexanic extract with a statistically significant difference.

As for the organic extracts, this reduction is much higher for ethanolic macerated (148.85 ± 0.43 mg TE/g E) and ethanolic extract (144.71 ± 0.35 mg TE/g E) with a statistically significant difference, followed by hexanic macerate, chloroformic macerate, chloroformic extract, and at the end hexanic extract, with values of 39.62 ± 0.08, 17.21 ± 0.10, 16.77 ± 0.69, and 9.53 ± 0.23 mg TE/g E, respectively; the organic extracts show a nonsignificant difference between them, except that the statistical difference is nonsignificant between chloroformic extract and chloroformic macerate (Table 7).

*(5) Reducing Power Assay (RP)*. The reducing power of organic extracts of *C. humilis* leaves is much higher than that of aqueous extracts. From the results obtained, we found that for aqueous extracts, the infused has the highest reducing power (2.495 ± 0.01 mg EAA/g E) followed by the decocted (2.46 ± 0.04 mg EAA/g E) and aqueous macerated (0.31 ± 0.007 mg EAA/g E) with a statistically insignificant difference between the three extracts.

Regarding the organic extracts, the ethanolic macerated presents the highest iron reduction capacity (10.86 ± 0.01 mg EAA/g E), followed by the ethanolic extract (10.14 ± 0.04 mg EAA/g E) with a statistically significant difference; nevertheless, the chloroformic and hexanic macerates and the chloroformic extract and the hexanic extract present low reducing powers with values of (2.12 ± 0.05, 1.41 ± 0.02, 1.14 ± 0.05, and 0.92 ± 0.07 mg EAA/g E) with a statistically significant difference between chloroformic and hexanic macerates and a statistically nonsignificant difference between chloroformic and hexanic extracts (Table 7).

The decocted and infused showed higher reducing power than the extracts: chloroformic and hexanic prepared hot by Soxhlet and chloroformic and hexanic macerated with a statistically significant difference.

#### 3.3.8. Antibacterial Activity

*(1) Agar Diffusion Method*. The disc diffusion method allowed highlighting the antibacterial power of the organic extracts of *C. humilis* on the selected strains which is translated by the appearance of inhibition zones. Extracts with inhibition zones greater than 15 mm are considered to possess strong antibacterial power; 8 to 15 mm are moderate, and inhibition zones of 1 to 8 mm represent weak antimicrobial activities [68]. The results are shown in Table 8.

The antibacterial activity of the organic extracts of the leaves of *C. humilis* towards 6 bacterial strains was tested by the diffusion method in agar medium. After 24 hours of incubation, the diameters of the inhibition zones around the disc were read and the results obtained are presented in Table 8.

Ethanolic extract showed moderate inhibitory activity against the following strains: *Proteus mirabilis* and *Listeria innocua* CECT 4030 with an inhibition diameters of 12 and 8.5 mm, respectively, and 8 mm was recorded for *Escherichia coli*, *Pseudomonas aeruginosa* CECT 118, *Staphylococcus aureus* CECT 976, and *Bacillus subtilis* DSM 6633 strains. The ethanolic macerated exhibited strong antimicrobial activity against *Proteus mirabilis* with an inhibition diameter of 16 mm at a concentration of 80 mg/ml and moderate inhibitory activity against the strains: *Listeria innocua* CECT 4030 and *Bacillus subtilis* DSM 6633 with an inhibition diameter of 14 mm at a concentration of 100 mg/ml; ethanolic macerated showed moderate activity against *Escherichia coli*, *Pseudomonas aeruginosa* CECT 118, and *Staphylococcus aureus* CECT 976 strains reflected by an inhibition diameter of 8 mm at concentration 100 mg/ml. Chloroformic extract showed moderate antimicrobial activity on *Proteus mirabilis* (10 mm), *Escherichia coli* (8 mm), *Pseudomonas aeruginosa* CECT 118 (8 mm), *Staphylococcus aureus* CECT 976 (8 mm), *Listeria innocua* CECT 4030 (8 mm), and *Bacillus subtilis* DSM 6633 (8 mm) at 100 mg/ml. Hexanic macerate showed moderate inhibitory power on the six strains tested: *Proteus mirabilis* (9 mm), *Listeria innocua* CECT 4030 (9 mm), *Pseudomonas aeruginosa* CECT 118 (8 mm), *Staphylococcus aureus* CECT 976 (8 mm), *Bacillus subtilis* DSM 6633 (8 mm), and *Escherichia coli* (7 mm) at 100 mg/ml. Chloroformic macerate and hexane extract showed no inhibition against the tested strains.

*(2) Determination of the Minimum Inhibitory Concentration (MIC) and Minimum Bactericidal Concentration (MBC) of Organic Extracts of C. humilis Leaves*. The MIC and MBC were determined only for the most active extracts found during the evaluation of antibacterial activity by the disc diffusion method; these concentrations will allow to determine the nature of the antibacterial activity: bacteriostatic or bactericidal.

The results and ratios of MIC and MBC are mentioned in Table 9. The ethanolic extract showed a low MIC value in the range of 5 mg/ml for *Escherichia coli* and *Listeria innocua* CECT 4030; *Pseudomonas aeruginosa* CECT 118 had a MIC value of 10 mg/ml; *Proteus mirabilis* and *Staphylococcus aureus* CECT 976 showed a MIC value in the range of 20 mg/ml; the highest MIC was obtained by *Bacillus subtilis* of 40 mg/ml. For the ethanolic macerated, the lowest MIC was 2.5 mg/ml recorded for the strains: *Escherichia coli*, *Pseudomonas aeruginosa* CECT 118, and *Listeria innocua* CECT 4030. *Bacillus subtilis* strain DSM 6633 had a MIC value of 5 mg/ml; *Proteus mirabilis* and *Escherichia coli* presented a MIC value of 10 mg/ml. The chloroform extract had the lowest MIC value of 1.25 mg/ml for *Listeria innocua* CECT 4030, followed by an MIC value of 5 mg/ml for *Bacillus subtilis* DSM 6633 and 10 mg/ml for *Proteus mirabilis* and for *Pseudomonas aeruginosa* CECT 118. *Escherichia coli* and *Staphylococcus aureus CECT 976* had MIC values of 20 and 40 mg/ml, respectively. Regarding hexane macerate, the lowest MIC value was obtained with *Listeria innocua* CECT 4030 (2.5 mg/ml), followed by *Pseudomonas aeruginosa* CECT 118, *Escherichia coli*, *Proteus mirabilis*, *Staphylococcus aureus* CECT 976, and *Bacillus subtilis* DSM 6633 with MIC values of 5, 10, 10, 20, and 20 mg/ml, respectively.

According to Table 9, the ratios of MBC/MIC indicated are between 2 and 32 mg/ml; we can deduce that our extracts have both bactericidal and bacteriostatic power on the six tested strains.

The MBC/MIC ratio indicates that the ethanolic extract presents a bactericidal activity against *Proteus mirabilis*, *Pseudomonas aeruginosa* CECT 11, and *Staphylococcus aureus* CECT 976 with values of 2, 4, and 4 mg/ml, respectively; on the other hand, this extract presents a bacteriostatic activity against *Listeria innocua* CECT 4030 (16 mg/ml). The ethanolic macerated has a bactericidal power on two tested strains: *Proteus mirabilis* and *Staphylococcus aureus* CECT 976 with a value of 4 mg/ml and a bacteriostatic effect against *Pseudomonas aeruginosa* CECT 11 and *Listeria innocua* CECT 4030 with a value of 16 mg/ml, while the *Escherichia coli* strain presents a resistance towards this same extract.

The chloroformic extract also has a bactericidal effect against *Staphylococcus aureus* CECT 976 and *E. coli* with 2 and 4 mg/ml, respectively, and a bacteriostatic power against *Proteus mirabilis* and *Pseudomonas aeruginosa* CECT 118 of 8 mg/ml. Hexanic macerate has a bactericidal effect against *Proteus mirabilis* (4 mg/ml), but *Listeria innocua* CECT 4030 seems to be resistant to this extract (32 mg/ml).

The results of the study of the antibacterial activity of the extracts of the leaves of *C. humilis* showed that the extracts have antimicrobial activities of varying degrees against the tested strains.

### 3.4. Principal Component Analysis (PCA)

The principal component analysis (PCA) allowed us to visualize the correlation between aqueous and organic extracts and their antioxidant capacity by the different tests used and the correlation between the activity of the extracts and their content in chemical compounds.

The PCA was carried out on nine individuals which are divided into three aqueous extracts (decocted, infused, and macerated) and six organic extracts (ethanolic extract, ethanolic macerated, chloroformic extract, chloroformic macerated, hexanic extract, and hexanic macerated) of the leaves of *C. humilis*, and this is in relation to eight variables represented, on the one hand, by the content of chemical compounds (total polyphenols, flavonoids, and catechic tannins) and, on the other hand, by the five tests used for the evaluation of the antioxidant activity: H_2_O_2_, DPPH, ABTS, FRAP, and PR.

#### 3.4.1. Correlation Matrix

According to the principal component analysis (PCA), the two main axes (F1 and F2) describe 90.48% of the total variance of the observations. We can therefore conclude that the interpretations made from this PCA will be highly significant.

PCA showed that the DPPH test is highly positively correlated with the ABTS test (*r*^2^ = 0.9214) and the latter is highly positively correlated with the FRAP (*r*^2^ = 0.9341) and RP (*r*^2^ = 0.9104) tests. The FRAP test shows a strong positive correlation with the RP test (*r*^2^ = 0.9743). Regarding chemical composition, the total polyphenol content is highly positively correlated with all tests except H_2_O_2_ (DPPH *r*^2^ = 0.9418, ABTS *r*^2^ = 0.9779, FRAP *r*^2^ = 0.9644, and RP *r*^2^ = 0.9271). The flavonoid content was also strongly positively correlated with the test (DPPH *r*^2^ = 0.8897). In addition, catechic tannins are highly positively correlated with DPPH (*r*^2^ = 0.9753) and ABTS (*r*^2^ = 0.8843) tests. In addition, total polyphenols are highly positively correlated with the catechic tannin content (*r*^2^ = 0.8924) (Table 10).

### 3.5. Graphical Representation of the Principal Component Analysis (PCA)

Figure 9 shows the distribution of the 9 individuals (extracts) in three groups G1, G2, and G3:

Group 1 gathers the ethanolic extract and the ethanolic macerated and the chloroformic macerate; the first two extracts present the highest contents of total polyphenols and tannins; they also express a better antiradical activity by the DPPH and ABTS tests and a high reducing power by the FRAP and RP tests. Total polyphenols and tannins seem to play a crucial role in the antioxidant effect. Chloroformic macerate contains a high content of flavonoids and shows a relatively high antiradical activity with the DPPH test.

Group 2 contains chloroformic extract, hexanic extract, and hexanic macerate; the chloroformic extract has a medium content of tannins; moreover, the hexanic extract and the hexanic macerate are moderately rich in flavonoids. These extracts present low antioxidant activity compared to the other organic extracts.

Group 3 includes the aqueous extracts: decocted, infused, and macerated which express low contents of phenolic compounds and a reduced antioxidant activity with all the tests except for the decocted which presents a notable activity via the test of H_2_O_2_ (Figure 9).

## 4. Discussion

### 4.1. Ethnopharmacological Survey

According to the results of the ethnopharmacological survey conducted on the species *C. humilis*, the average age of the respondents is 50.47 years; the evolution of the use of the plant in traditional medicine with age can be explained by the fact of the accumulation of experience and traditional phytotherapeutic knowledge with age. These results are similar to those advanced by Medjati in Algeria who found that the frequency of use of *C. humilis* in the medicinal field increases with the age of the respondents; people over 60 years old have the highest percentage of use (100%) [16].

For the percentage of use of the species in traditional medicine, it is very close between women (84.21%) and men (90.27%); our results corroborate with the ethnobotanical works carried out in Algeria on the same species with a very close percentage; it is 80% for women and 84.71% for men [16]. This is not the case for studies that have shown that ethnobotanical knowledge related to other species varies mostly with gender; the work conducted by Boulfia and his collaborators in the same area of the present study showed that men use medicinal plants more frequently than women [5, 6]. Another ethnobotanical study conducted in Morocco by Mehdioui and Kahouadji whose aim is at describing the different uses of medicinal plants in one of the communes of the province of Essaouira showed that women have more knowledge about medicinal species compared to men (53% versus 47%) [69]. In other ethnobotanical studies conducted in northern Morocco, the first was done to identify medicinal plants used in the treatment of diabetes and hypertension, among the population living in the forest of Izarène in northern Morocco, which revealed that it is women who use medicinal plants much more than men (74.36% against 25.64%) [70]; the second conducted in Mechra Bel Ksiri on medicinal plants used in traditional medicine in the treatment of urinary tract infections showed that women use medicinal plants much more (87%) than men (61.90) [71]. An ethnobotanical survey was conducted in the region of Rabat-Sale-Kenitra on the plants used for the treatment of chronic diseases and showed that women have a good knowledge of traditional medicine than men, with a frequency of 59.05% against 40.94% for men [72].

According to the data obtained, illiterate people use medicinal plants much more to treat their illnesses (65.27%), which could be explained by the high cost of treatments offered by modern medicine, which are the limits that can justify this recourse to traditional pharmacopoeia, also because illiterate people are the oldest and have much more information about medicinal plants, since this segment of the population of respondents holds much of the ancestral knowledge that is part of the oral tradition. Leonti assumes that illiterate societies generally transmit cultural knowledge orally in a vertical fashion [73]. Ribeiro and collaborators also found that 75% of respondents acquired their knowledge of plant use from family tradition in an ethnobotanical survey conducted in Brazil [74]. Similarly, the respondents stated that the therapeutic recommendations on the plant in question are made by their grandfathers and grandmothers, which means vertically.

The results obtained with people with a higher level of education can be explained by the fact that they are aware of the toxicity caused by the misuse of medicinal plants. Our results corroborate with other ethnobotanical surveys done at the national level such as an ethnobotanical study conducted in the High Moulouya which proved that the dominant users of traditional medicine are illiterate people with a percentage of 41% [75]. Our results are also in agreement with other studies and ethnobotanical surveys conducted in Algeria such as Medjati who found that there is a correlation between the level of study and the medicinal use of *Chamaerops humilis* between illiterate people, primary-level people, secondary-level people, and university-level people with percentages of 96.7%, 89.2%, 83%, and 58.9%, respectively, [16]. Other studies were conducted nationwide, such as that of Mehdioui and Kahouadji who showed that the vast majority of users of medicinal plants are illiterate, with a percentage of 66% followed by people with a primary level with 26%, while those with secondary and university levels of education use very little medicinal plants (secondary 7%, university 1%) [69]. Hmamouchi and his collaborators conducted a study on the traditional practices of using Moroccan medicinal plants in rheumatology; in this study, they found that there is a positive correlation between the level of study and the percentage of use of medicinal plants (illiterate 53%, secondary 19%, and university 4%) [76].

According to the results of the survey, we found that the names attributed to *C. humilis* and its different parts vary according to the dialect of the respondent (Arabic/Amazigh). In this sense, studies carried out in Morocco have reported that *C. humilis* is called “Dûm” in the region of Taounat [77]. In the region of Sidi Bennour, the whole plant is also called “Eddoum” and the fruit “Lghaz” [78]. In the Middle Atlas of Morocco, the palm heart has a different name; it is called “Jmakh” [79]. In Algeria, the whole plant takes a similar name to that in Morocco; it is called “Doum” [16, 80].

The heart of palm and spadices are the most used parts by the population of the region of Taza (79.49%). These results are consistent with those obtained by Medjati and collaborators Okkacha and collaborators who showed that the most used parts in Algeria are the heart of palm and spadices [16, 18].

The survey allowed us to list a number of chronic diseases treated by the heart of palm: digestive disorders, cardiovascular system disorders, respiratory system disorders, diabetes, hepatitis, hair loss, and weakening of the immune system. Our results are consistent with those of a survey conducted in the province of Taounate which showed that the fruits in decoction are used as a treatment for liver disorders, gallstones, and against diabetes [77]. Another study conducted in the Moroccan central plateau with the objective of describing the medicinal plants used in the treatment of dermatological conditions indicated that the fruits of *Chamaerops humilis* are used against digestive disorders [81].

In Algeria, according to a survey conducted by Medjati et al., the heart of palm and spadices are used against gastrointestinal diseases and the fruits as antiseptic, the roots are used in decoction against intestinal worms and as a treatment for anemia, they are also used in women for cleaning the uterus after childbirth, and the leaves are used against gastrointestinal attacks and hepatitis [16].

Okkacha and his collaborators also demonstrated from a survey conducted in Algeria that the heart of palm is used against bloating, gastric pain, and constipation, while spadices are used as a tonic; on the other hand, the therapeutic use of the fruits of *Chamaerops humilis* is not reported by the respondents; on the other hand, the leaves of *Chamaerops humilis* are used for the treatment of diabetes [18].

The heart of palm and spadices are generally consumed raw without preparation (95.38%); this could be explained by the abundance of this plant in the region; the heart of palm is considered the fruit of the season, and it is sold everywhere in the province of Taza, which is in agreement with the results obtained by two studies conducted in Algeria by Medjati et al. and by Okkacha and his collaborators who found that the heart palm is consumed raw in salad. The fruits are also used raw with a percentage of 59.32% or in association with pure honey or olive oil (38.98%) and weakly used in decoction (1.69%). This use can be explained by the synergic effect of this part with the honey or the olive oil (Figure 8). On the other hand, the decoction dominates as a mode of preparation for the roots (90.90%), the infusion mode is less used among the respondents with 9.09% (Figure 8), and the surveyed population thinks more about the decoction because it allows to warm the body and to disinfect the roots which are in direct contact with the soil to eliminate the toxic effect of some recipes. During our survey, we clearly found that only the leaves in the fresh state are used after grinding (47.82%), decoction (34.78%), and maceration (17.39%). For Okkacha and his collaborators, the leaves are used much more in maceration; in addition, Medjati et al. showed that the leaves are used in maceration or else in decoction [16, 18]. These same surveys did not indicate the use of one or more parts in combination with other substances.

*C. humilis* has several uses other than being medicinal: food for humans (heart of palm, spadice, and fruit), food for animals (leaves and fruit), handicraft use (leaves), and tool for dishes (leaves), and the whole plant is used as firewood. These results confirm the results of other work done on the same species; Guarrera and Savo conducted a study on the traditional use of wild food plants in Italy; they found that the bud of *Chamaerops humilis* was consumed as a salad in Sicily [82]. Other ethnobotanical studies conducted on *Chamaerops humilis* in Algeria by Okkacha and collaborators in 2011 found that heart of palm, spadice, and leaves are used for therapeutic purposes [18], while Medjati et al. showed that all parts of the plant are used therapeutically [16].

### 4.2. Mineralogical Composition of *C. humilis* Leaves

Mineralogical analysis shows that leaves of *C. humilis* constitute a resource of minerals, with a high content of iron, potassium, phosphorus, and magnesium, in addition to significant quantities of sodium, copper, and zinc. Calcium and strontium are present at low levels. Iron is a fundamental constituent for plants and a vital element of hemoglobin; it also plays an important role in DNA synthesis and electron transport. However, if the concentration of iron exceeds this limit, the ingestion of these plants can lead to the accumulation of iron in the human body [37]. In addition, the analyzed part has significant contents of elements K, Ca, Cu, and Zn which are responsible for insulin secretion by islet beta cells and are involved in the potentiation of insulin action [83]; this could be due to their antioxidant effect. The results also show that the studied part is rich in magnesium that is an essential mineral for the human body; it is necessary for the synthesis of ATP, proteins, bone structure, stabilization of membranes, and metabolism of blood sugar and also intervenes in the functioning of many enzymatic systems at the level of the human body. Sodium in turn is an important component in the regulation of osmotic balance of all intra/intercellular fluids [84]. Selenium in turn at low doses is capable of blocking free radical synthesis [85]. In addition, according to Kolachi and colleagues, selenium can reduce the incidence of cancer and associated mortality in humans [86]. According to Pilmane and colleagues, strontium has a dual action on bones: it is able to improve bone formation and slow bone resorption [87].

The leaves of *C. humilis* provide a source of minerals that is likely responsible for its biological activities; according to Grela and colleagues, the antioxidant activity was attributed to mineral components such as copper, manganese, and iron [88]. A study by Pandya found that low doses of trace minerals such as Cu and Zn inhibit the production of oxidative free radicals [85]. In addition, mineral imbalance would change the content of flavonoids considered as the proven antioxidant compound [89]. Our recent study conducted on *Haloxylon scoparium* had shown that the high antioxidant capacity of aqueous and organic extracts of this plant is correlated and explained by its richness in Fe (60909.00), K (27452.10), Mg (10059.90), P (1125.39), Na (1054.65), and Cu (438.93 mg/kg) [43].

Studies conducted on plants collected in the region of Taza, Morocco, have also revealed the richness of the said plants in mineral elements that are involved in their biological properties: *Juglans regia* has a high level of Fe (19849.8), K (3487.8), Mg (2631.03), and P (691.02 mg/kg), *Leopoldia comosa* is rich in Fe (33552), K (1843.14), P (756.36), Na (439.65), Cu (303.9), Mg (272.37), and Ca (20.55 mg/kg), and *Ajuga iva* has contents of 112.00 mg/l Fe, 44.071 mg/l K, and 16.572 mg/l Na [44, 90, 91].

### 4.3. Phytochemical Study of the Leaves of *C. humilis*

#### 4.3.1. The Yield of the Extractions

The phytochemical study carried out on the leaves of *C. humilis* revealed that the best yield was obtained with the most polar solvents and that the yields of hot extractions are higher than those obtained cold. The yield of the extraction varies according to the plant species, the part used in the extraction, the period of harvest of the plant, the type of soil, the climate, the geographical position, the conditions of drying in particular the duration, the form of the plant material (powder or fragments), the nature of the solvent used in the extraction and its polarity, and the conditions of extraction (temperature, duration of extraction, and ratio solvent/plant material).

According to Mylonaki and collaborators, the concentration of ethanol and the duration of extraction influence the extraction yield of *Olea europaea* [92]. Similarly, Wu and colleagues found that temperature, extraction time, and solvent to plant material ratio affect the yield of *Ziziphus jujuba* [93].

Studies conducted in our laboratory under the same experimental conditions as the present study show that the part of the plant, the choice of solvent, the extraction modality (aqueous or organic), and the temperature (hot or cold extraction by maceration) influence the extraction yields, the contents of secondary metabolites of the extracts, and consequently their biological activities. Indeed, Bouabid and her collaborators reported that the best yields are obtained with polar solvents and hot extraction gives the best yields compared to cold extractions of the underground part of *Atractylis gummifera* [46, 58]. Senhaji and her collaborators found that the aqueous macerate and the methanolic extract prepared hot from the aerial part of *Ajuga iva* have the highest yield of 13.31 and 9%, respectively. Similarly, the aqueous macerate and methanolic extract of the aerial part of *Anabasis aretioides* show the best yield of 3.41 and 3.39%, respectively, [47, 48]. Boulfia and his collaborators found that ethanolic extract and decocted of *Juglans regia* have the highest yields of 22.04 and 14%, respectively [49]. In addition, the highest yield was obtained by the decocted prepared from *Leopoldia comosa* [44]. Another study recently conducted on *Haloxylon scoparium* showed that the two extracts were prepared under heat and with the most polar solvents (water and methanol): the decocted and the methanolic extract show the highest yields of 16, 8, and 14.35% [43].

#### 4.3.2. Extraction by Hydrodistillation

The extraction by hydrodistillation of essential oils from the leaves of *Chamaerops humilis* var. argentea André has given only a few traces whose calculation of the yield has been infeasible. Works were carried out on the same species with the technique of hydrodistillation but in different geographical locations whose results obtained are also variable. Indeed, Okkacha and his collaborators in Algeria reported that extraction of essential oils from *Chamaerops humilis* leaves yielded only trace amounts of essential oil, while in Morocco, Khoudali and his collaborators found that extraction of essential oils from *Chamaerops humilis* leaves produced 0.19% [15, 94].

Several factors can affect the extraction of essential oils in the same species including the season and area of harvest, the stage of growth, the method of extraction, and the condition of the plant material spawned or dried. According to Ranjitha and Vijiyalakshmi, among all the extraction methods, the supercritical carbon dioxide method is the most effective method for extraction of essential oils [95].

#### 4.3.3. Phytochemical Screening

Phytochemical screening carried out on both the leaf powder and the aqueous and organic extracts prepared from them showed that the plant material of the studied part contains sterols, saponins, flavonoids, free quinones, and catechic tannins. The ethanolic extract, ethanolic macerated, decocted, and infused possess flavonoids, saponins, quinones, and catechic tannins. Sterols are present only in the hexanic extract and the hexanic macerate. Alkaloids are absent in all extracts and in the powder of the studied plant part.

The complete study of the phytochemical screening highlights the presence of chemical compounds with interesting biological activities. The presence of tannins, endowed with tissue renewal properties, is powerful in the healing process of wounds due to diabetes, flavonoids possess antioxidant properties, and they could be used to prevent atherosclerosis [96]. The therapeutic effects of the leaves of *C. humilis* against digestive disorders in cattle are produced by different chemical compounds which are sterols, total polyphenols, flavonoids, catechic tannins, and quinones. The presence of these compounds in this part would justify its use in the traditional pharmacopoeia.

The phytochemical study reported by Benmehdi and collaborators showed that the aqueous, methanolic, and diethyl ether extracts of saw palmetto leaves contained the gall tannins, while the catechic tannins were absent in all the extracts studied [17]; another phytochemical study done on the methanolic extract of the leaves showed the presence of tannins, flavonoids, quinones, and saponins [97]. Khoudali and his collaborators found that the methanolic extract of *Chamaerops humilis* leaves contains both gallic and catechic tannins [15].

Under the same operating conditions, a work conducted in our SNAMOPEQ on plants from the same region as *C. humilis* states that phytochemical screening revealed the presence of catechic tannins, saponins, and sterols in the aerial part of *Anabasis aretioides* [47]; the underground part of *Atractylis gummifera* is rich in catechic tannins and flavonoids [46]. *Juglans regia* is rich in catechic tannins, flavonoids, anthraquinones, and free quinones; *Leopoldia comosa* has catechic tannins, flavonoids, and free quinones [44, 49]. The aerial part of *Ajuga iva* contains catechic tannins, flavonoids, saponins, and sterols [48].

#### 4.3.4. Determination of Total Polyphenols, Flavonoids, and Catechic Tannins Contents

Phenolic compounds are more abundant in the organic extracts compared to the aqueous extracts. For the latter, the decocted presents the highest content of total polyphenols (13.23 ± 0.19 mg EAG/g E), flavonoids (56.36 ± 0.39 mg EQ/g E), and tannins (10.08 ± 0.07 mg EC/g E). These results show that high temperature allows a better extraction of total polyphenols, flavonoids, and catechic tannins. For organic extracts, ethanolic macerated and ethanolic extracts were richer in total polyphenols (100.27 ± 0.66; 96.99 ± 0.82 mg EAG/g E) and tannins (52.11 ± 0.24; 50.27 ± 0.99 mg EC/g E) with a nonsignificant difference. For flavonoids, chloroformic macerate contains the highest flavonoid content (542.7 ± 24.03 mg EQ/g E), followed by ethanolic macerated which also has high flavonoid content with a significant difference with chloroformic macerate. From these results, it is deduced that the phenolic content in the extracts examined depends on the polarity of the solvent used and the method of extraction; Dary and collaborators conducted an extraction optimization study of three bioactive alkaloids: palmatine, roemerine, and tetrahydropalmatine from *Stephania cambodica* tuber; they found that microwave-assisted extraction (MAE) was more efficient than ultrasonic-assisted extraction (UAE) for the extraction of tetrahydropalmatine but UAE increased the yield of palmatine and roemerine. In addition, the liquid-to-solid ratio, percentage of solvent, and extraction time also influenced the extraction of these three alkaloids [98].

A study made in Algeria by Benahmed and collaborators revealed that the cold-prepared methanolic macerated of *Chamaerops humilis* leaves presents a value of 26.8 ± 0.41 mg/g in polyphenols and 40.7 mg EC/g E in flavonoids; these values are still low compared to the content of total polyphenols (100.27 ± 0.66 mg EAG/g E) and flavonoids (468.25 ± 9.07 mg EQ/g E) obtained in our study. Similarly, for a study conducted in Morocco, Khoudali and colleagues quantified polyphenols (99.8 mg EAG/g E) and flavonoids (3.70 mg EQ/g E) at the level of methanolic extract of leaves of the same species [15]. These values remain low compared to those of the ethanolic and ethanolic macerated extract determined in our present study. This quantitative difference is due to several factors related to the variety; in our study, we worked on the variety argentea, part of the plant, place, and stage of harvest of the plant and also to the experimental conditions that we adopted for our study: choice of extraction solvents, modalities of lime and cold, and aqueous and organic extractions. Studies carried out on plants from the region of Taza, Morocco, under the same experimental conditions by Senhaji and his collaborators confirm these findings. Indeed, the decocted and aqueous macerate of the aerial part of *Anabasis aretioides* present high contents of total polyphenols (1.78 ± 0.003; 0.92 ± 0.03 mg EAG/g E); moreover, ethyl acetate is the recommended solvent for the extraction of total polyphenols [47]. Another study conducted on the underground part of *Atractylis gummifera* revealed that the methanolic macerated is richer in total polyphenols (102.88 ± 1.38 mg EAG/g E), flavonoids (17.25 ± 0.06 mg ER/g E), and tannins (144.09 ± 3.96 mg EC/g E) [58]. According to Senhaji and collaborators, decoction is the mode that allows high extraction of total polyphenols (3.75 ± 0.02 EAG/g E), flavonoids (22.40 ± 0.36 mg ER/g E), and tannins (15.49 ± 0.17 mg EC/g E) from the aerial part of *Ajuga iva* [48]. Boulfia and collaborators found that the acetone macerate of *Juglans regia* contained the highest content of phenolic compounds (327.972 ± 0.06 *μ*g EAG/mg E), flavonoids (1267.981 ± 2.911 *μ*g EQ/mg E), and catechic tannins (38.056 ± 1.886 *μ*g EC/g E). In addition, the diethyl ether extract prepared from *Leopoldia comosa* bulb contains high content of total polyphenols (129.75 ± 0.29 *μ*g EAG/mg E), flavonoids (988.26 ± 0.18 *μ*g EQ/mg E), and tannins (30.22 ± 0.15 *μ*g EC/g E) [44, 49]. Our recent study done on *Haloxylon scoparium* revealed that the methanolic extract is rich in total polyphenols (161.65 ± 1.52 *μ*g EAG/mg E) and catechic tannins are abundant in the ethyl acetate extract (23.69 ± 0.6 *μ*g EC/mg E); the decocted also has a high flavonoid content (306.59 ± 4.35 *μ*g EQ/mg E) [43].

The catechic tannins contained at the level of medicinal plants also present therapeutic virtues. According to Zahoui et al., the catechic tannins present at the level of the leaves of *Combretum micranthum* give it a powerful diuretic power [99] and anti-inflammatory properties, thanks to its astringent character; the tannins can contribute to the treatment of acute diarrhea [100], which confirms the use of the leaves of *C. humilis* to treat problems of the digestive system. The existence of sterols in the studied plant part confirms its use in traditional medicine as an antimicrobial agent. According to a study done by Geethalakshmi and Sarada, sterols isolated from *Trianthema decandra* L. possess antimicrobial activity *in vitro* against Gram-positive and Gram-negative bacteria [101].

#### 4.3.5. Antioxidant Activity

In this study, we noticed that the decocted has the highest antioxidant capacity for DPPH, ABTS, H_2_O_2_, and FRAP tests in comparison with the infused and aqueous macerated. This same extract has a higher scavenging capacity than the reference standard: ascorbic acid (14.35 ± 0.002) in the H_2_O_2_ test. For the reducing power (RP) test, we notice that the infused and decocted extracts have a better reducing power with a statistically nonsignificant difference between these two aqueous extracts. The evaluation of the antiradical and antioxidant activities of the organic extracts reveals that the ethanolic macerated presents the highest activity for the five tests used: DPPH (CI 50 = 31.18 ± 0.66 *μ*g/ml), ABTS (108.28 ± 1.29 mg ET/g E), H_2_O_2_ (37.34 ± 0.55%), FRAP (148.85 ± 0.4323 mg ET/g E), and RP (10.86 ± 0.01 mg EAA/g E). In addition, the ethanolic macerated shows a significantly higher percentage of inhibition than the reference standard for the H_2_O_2_ test. This extract also shows a statistically insignificant difference with the ethanolic extract prepared at hot Soxhlet for both H_2_O_2_ (36.51 ± 0.33%) and DPPH (IC 50 = 44.25 ± 2.31 *μ*g/ml) tests and with the chloroformic macerate for the H_2_O_2_ test (35.79 ± 0.29%).

These results show that the leaves of *C. humilis* are endowed with a remarkable antioxidant power, which could explain the use of this part in phytotherapy to solve digestive problems. Indeed, numerous scientific researches have pointed out the link between reactive oxygen species (ROS) and digestive pathologies; free radicals are involved in many human gastrointestinal diseases such as gastritis, hepatitis (e.g., infectious and toxic etiologies), inflammatory bowel diseases, and digestive cancers [102, 103].

In comparison within the same species and the same studied part, our results of the DPPH antiradical activity are not very close to those obtained in Morocco by Khoudali and his collaborators, on the methanolic extract with an IC_50_ = 24.5 *μ*g/ml. On the other hand, our ethanolic extracts show a higher capacity to trap the radical than those obtained by Benahmed and collaborators for the methanolic extract (IC_50_ = 180.71 *μ*g/ml) prepared from Algerian *Chamaerops humilis* leaves and by Gonçalves and collaborators on the methanolic macerated of *Chamaerops humilis* leaves harvested in Portugal (IC_50_ = 346 *μ*g/ml) [15, 97, 104]. This variation is due to the geographical area, harvesting season, preparation form, and temperature and extraction time adopted for each study.

The reducing power of *C. humilis* is probably due to the existence of the hydroxyl group in phenolic compounds that can be like an electron donor. Because of this, antioxidants are considered to be reducers and inactivators of oxidants [105]. Gonçalves and collaborators tested the reducing power of methanolic extract of *Chamaerops humilis* leaves harvested from Algare, a region in the south of Portugal; they found that they present a value of 434.34 ± 13.71 *μ*mol/g E [104]. Under the same operative conditions as in our study, a phytochemical study conducted by Bouabid and collaborators showed that the methanolic macerate of the underground part of *Atractylis gummifera* L. presents the most expressed antioxidant activity for the H_2_O_2_ test (19.24 ± 1.102%), ABTS (122.6 ± 0.63 mg TE/g E), FRAP (102.5 ± 1.66 mg TE/g E), and RP (96.15 ± 1.12 mg EAA/g E) [58]. In addition, Senhaji and her collaborators conducted a phytochemical study on the aerial part of *Ajuga iva* subsp.; they found that the decocted had a strong reducing power compared to the infused and aqueous macerate for FRAP and RP tests [91]. Another phytochemical study conducted on the aerial part of *Anabasis aretioides* showed that the methanolic macerated exhibited the highest antioxidant activity for all four assays: DPPH (IC_50_ = 52.91 ± 0.24 *μ*g/ml), ABTS (48.99 ± 1.316 *μ*g TE/mg E), FRAP (99.73 ± 3.570 *μ*g TE/mg E), and RP (72.176 ± 0.540 *μ*g AAE/mg E) [47]. Boulfia and his collaborators found that the best antioxidant activity of *Juglans regia* bark was obtained with the acetone macerate which was found to be the most active according to the five different tests: H_2_O_2_ (24.13 ± 1.81%), DPPH (IC_50_ = 5.573 *μ*g/ml), ABTS (602.29 ± 0.34 *μ*g ET/mg E), FRAP (759.11 ± 0.27 *μ*g TE/mg E), and RP (685.68 ± 0.82 *μ*g AAE/mg E); the diethyl ether extract of *Leopoldia comosa* also showed antioxidant power via the same tests: H_2_O_2_ (62.67 ± 0.06%), DPPH (IC_50_ = 10.08 ± 0.01 *μ*g/ml), ABTS (381.63 ± 0.63 *μ*g ET/mg E), FRAP (394.77 ± 0.74 *μ*g TE/mg E), and RP (356.7 ± 0.92 *μ*g AAE/mg E) [44, 49]. Evaluation of the antioxidant activity of the methanolic extract of the aerial part of *Haloxylon scoparium* showed a high antioxidant capacity compared to the other extracts tested: H_2_O_2_ (20.91 ± 0.27%), DPPH (IC_50_ = 39.63 ± 2.03 *μ*g/ml), ABTS (50.75 ± 0.72 *μ*g ET/mg E), FRAP (163.37 ± 1.52 *μ*g TE/mg E), and RP (116.18 ± 8.19 ± 0.82 *μ*g AAE/mg E) [43].

The results obtained in the present study confirm the existence of a certain correlation between the content of phenolic compounds and the antiradical and antioxidant activities. In fact, the extract and ethanolic macerated prepared hot by Soxhlet and cold by maceration showed high contents of total polyphenols and were found to be the extracts with the highest antifree radical and antioxidant activity in the five tests used. Indeed, the antioxidant activity may be due to the inhibition of radical formation or the scavenging of the formed radicals [106]. Furthermore, mineral elements could also be responsible for the antioxidant capacity of *Chamaerops humilis*; a study conducted on *Phoenix dactylifera* fruits showed a strong correlation between antioxidant activity and mineral composition; the K content was strongly correlated with the FRAP test (*r*^2^ = 0.800) and with the H_2_O_2_ test (*r*^2^ = 0.889) [107]. From our mineralogical analysis, we found that *C. humilis* leaves are rich in potassium (9354.90 mg·kg^−1^ dry matter) which might be responsible for its antioxidant power. In addition, several works have announced the contribution of minerals as antioxidant elements. For Grela and collaborators, the antioxidant activity is due to mineral compounds such as copper, manganese, and iron [88].

#### 4.3.6. Antibacterial Activity

The results of the study of the antibacterial activity of the extracts of the leaves of *C. humilis* show that the extracts have antimicrobial activities of varying degrees against the tested strains with inhibition diameters from 7 to 16 mm. The ethanolic macerated shows the highest inhibition against *Proteus mirabilis* with an inhibition diameter of 16 mm at 80 mg/ml and medium inhibition against *Bacillus subtilis* DSM 6633 and *Listeria innocua* CECT 4030 with a zone of 14 mm at 100 mg/ml. This is in agreement with the high amount of polyphenols contained in this extract (100.27 ± 1.95 mg EAG/g E) and tannins (52.11 ± 1.02 mg EC/g E).

Ethanolic and chloroformic extracts showed moderate inhibition against *Proteus mirabilis* of 11 mm and 10 mm, respectively, at 100 mg/ml. The ethanolic extract contains the saponins and coumarins, compounds with antimicrobial action; a work by Abd El-Fattah and collaborators confirmed the antibacterial effect of synthetic coumarin derivatives against *B. Subtilis* (28 mm), *P. Aeruginosa* (22 mm), and *E. Coli* (24 mm) [108]. In addition, Dong and collaborators reported that saponin “-O-*β*-D-glucopyranosyl-(1→3)-*α*-larabinopyranosyl-phytolaccagenic acid-27-oxo-28-O-*β*-D-glucopyranosyl” extracted from *Chenopodium quinoa* Willd had an inhibitory effect on the growth of *S. aureus* (11.70 mm) [109].

Hexanic macerate had a moderate inhibitory effect against *Proteus mirabilis*, *Listeria innocua* CECT 4030, and *Bacillus subtilis* DSM 6633 with a zone of 9, 9, and 8 mm, respectively, at 100 mg/ml. From phytochemical screening, we found that this extract contains sterols which are probably responsible for this antimicrobial action. A study conducted by Geethalakshmi and Sarada shows that sterols isolated from the leaves of *T. decandra* had a growth inhibitory action against *Staphylococcus aureus* MTCC 29213 (20 mm), *Escherichia coli* MTCC 443 (23 mm), *Pseudomonas aeruginosa* MTCC 1035 (23 mm), and *Bacillus subtilis* MTCC 121 (22 mm) [101]. In addition, Nazarparvar and collaborators showed that n-butanol extract of *Nigella sativa* is rich in terpenoids and exhibited antimicrobial effect against *Pseudomonas aeruginosa*, *Klebsiella pneumoniae*, *Acinetobacter baumannii*, and *Yersinia enterocolitica* [110].

Based on the results reported in Table 9, the MBC/MIC ratio ranged from 2 to 32 mg/ml. The MBC/MIC ratio indicates that the ethanolic macerate had bactericidal power on two strains tested: *Proteus mirabilis* and *Staphylococcus aureus* CECT 976, and a bacteriostatic effect against *Pseudomonas aeruginosa* CECT 11 and *Listeria innocua* CECT 4030. The ethanolic extract showed bactericidal activity against *Proteus mirabilis*, *Pseudomonas aeruginosa* CECT 11, and *Staphylococcus aureus* CECT 976. According to Armbruster and collaborators, *Proteus mirabilis* is capable of causing various human infections, especially those of the gastrointestinal tract [111]; this explains the traditional use of *Chamaerops humilis* leaves by the population for the treatment of digestive system problems in livestock. This extract also exhibits bacteriostatic activity against *Listeria innocua* CECT 4030. The chloroformic extract prepared by hot Soxhlet also shows bactericidal effect against *Staphylococcus aureus* strain CECT 976 and *E. Coli* and a bacteriostatic power against *Pseudomonas aeruginosa* CECT 118 and *Proteus mirabilis*.

Under the same operating conditions as in the present study, the chloroform extract of the aerial part of *Anabasis aretioides* tested in our laboratory gave identical MIC value for *Pseudomonas aeruginosa*, *Staphylococcus aureus* CECT976, and *Bacillus subtilis* DSM 6633 strains in the range of 100 mg/ml and 50 mg/ml for *Escherichia coli* K12 and *Proteus mirabilis* [47]. Lamchouri and her collaborators reported that ethyl acetate extract of the aerial part of *Haloxylon scoparium* exhibits moderate antibacterial activity (7–12 mm) against *Staphylococcus aureus* strain [112]. In the present study, hexane macerate of *Chamaerops humilis* shows bactericidal effect against *Proteus mirabilis*; on the other hand, *Listeria innocua* CECT 4030 seems to be resistant towards this extract. This activity could be explained by the nature of the antimicrobial molecules extracted and soluble in the hexanic macerate. Indeed, the phytochemical screening mentioned the presence of sterols which may be responsible for the inhibition of *Proteus mirabilis*. In this sense, Singh and collaborators found that the highest antibacterial capacity was observed for sterols in *E. hirta* fruits (21 mm) [113]. In addition, studies conducted on plants from Taza region reported that *Ajuga iva* had the highest inhibition diameter for petroleum ether extract against *Proteus mirabilis* strain (14 mm) [91]; *Juglans regia* acetone macerate was found to be the most active with an inhibition diameter of 17 and 18 mm against *Proteus mirabilis* and *Pseudomonas aeruginosa* [90].

### 4.4. Principal Component Analysis (PCA)

According to the principal component analysis, the DPPH, ABTS, FRAP, and RP tests used for the evaluation of antioxidant activity are highly correlated with each other: DPPH with ABTS (*r*^2^ = 0.92), ABTS with FRAP (*r*^2^ = 0.93), ABTS with RP (*r*^2^ = 0.91), FRAP with RP (*r*^2^ = 0.97), and RP with ABTS (*r*^2^ = 0.91). Indeed, these correlations show that our extracts possess both a better scavenging power towards free radicals demonstrated by the tests (DPPH and ABTS) and also show a better Fe(III)-reducing capacity via the tests (FRAP, RP). This probably shows the presence in our extracts of antioxidant molecules that can intervene by two types of reaction mechanisms. The reactions involved may act according to the test used; for the FRAP and RP tests, it is a reduction of Fe (III), based on an electron transfer. Concerning the DPPH and ABTS tests, these two radicals can be neutralized either by direct reduction via electron transfer or by trapping the radical via a hydrogen atom transfer [114]. Regarding the H_2_O_2_ assay, it shows the lowest correlation to the other assays which could be explained by the nature of each oxidizing radical and its mechanism of action on antioxidant compounds; according to Winterbourn, hydrogen peroxide is a strong oxidant with two electrons but much of its two-electron oxidation reactions are too slow to be biologically interesting [115].

The content of polyphenols presents a high correlation with the results of the antioxidant activity obtained by the four tests: (ABTS *r*^2^ = 0.97), (FRAP *r*^2^ = 0.96), (DPPH *r*^2^ = 0.94), and (RP *r*^2^ = 0.92). Thus, the antioxidant activity of our extracts can be attributed to polyphenols which would be endowed with antioxidant effects. Indeed, according to the study conducted by Marimoutou and collaborators on medicinal plants *A. borbonica* and *D. apetalum* and *G. mauritiana*, extracts of the plants rich in polyphenols decreased the production of ROS and the secretion of the proinflammatory markers IL-6 and MCP-1 induced by the mediators H_2_O_2_, TNF*α*, and LPS. Such a protective action was associated with increased gene expression of the antioxidant enzyme superoxide dismutase and decreased mRNA levels of the proinflammatory transcription factor NF-*κ*B [116]. Flavonoids also show high correlation with DPPH (*r*^2^ = 0.88) and ABTS (*r*^2^ = 0.75) tests, which means that flavonoid compounds in our extracts possess much more antiradical power; in this sense, several researchers have reported the antioxidant effect of flavonoids [117, 118].

In addition, catechic tannins had a high correlation with DPPH (*r*^2^ = 0.97) and ABTS (*r*^2^ = 0.88), which indicates that tannins contained in the studied extracts are able to scavenge free radicals either by electron transfer or by hydrogen atom transfer, this is in agreement with what is announced in the literature by Okuda that tannins intervene by the antiradical mechanism for scavenging the DPPH free radical [119].

Through the results of the PCA, we note that polyphenols present a stronger correlation with tannins (*r*^2^ = 0.89) than flavonoids (*r*^2^ = 0.75); these results indicate that the polyphenols contained in the extracts of the leaves of *C. humilis* are mainly constituted by catechic tannins; these last ones could be responsible of the astringent taste of the plant. According to Gombau and colleagues, condensed and hydrolyzable tannins contribute to the astringency of wine [120].

Work conducted with other plants from the Taza region and reported by Boulfia and collaborators reveals that phenolic compounds, flavonoids, and tannins are strongly correlated with the antioxidant activity of *Juglans regia* and *Leopoldia comosa* [44, 49]. In addition, Senhaji and her collaborators demonstrated a good correlation between the total polyphenol content and DPPH, ABTS, FRAP, and RP tests performed on *Anabasis aretioides*. A positive correlation was also found between the polyphenol contents of *Ajuga iva* and the antioxidant capacity assessed by the ABTS test [47, 48].

## 5. Conclusion

The ethnopharmacological survey conducted among the population of the province of Taza has allowed us to know the frequent uses of different parts of the plant *C. humilis* by the local population to cure many diseases and ailments. According to the results of the survey, the diseases of the digestive system are the most treated by the different parts of the plant in question.

According to the mineralogical analysis, the leaves of *C. humilis* present an excellent source of minerals with therapeutic and pharmacological properties including Fe, K, P, Mg, Na, Cu, Ca, and Zn.

The quantitative analysis carried out revealed that the aqueous and organic extracts of the plant have highly elevated contents of total polyphenols, flavonoids, and tannins. All these compounds are endowed with a great therapeutic power.

The evaluation of the antioxidant activity of the aqueous and organic extracts of the leaves of *C. humilis* determined by five methods (DPPH, ABTS, H_2_O_2_, FRAP, and PR) showed that this part of the plant possesses potent antioxidant and antiradical activities, probably attributable to the chemical and mineral compounds that it contains.

The principal component analysis showed the presence of a strong positive correlation, on the one hand, between the four tests used for the study of the antioxidant activity of ABTS, DPPH, FRAP, and RP and, on the other hand, between these tests and the composition in total polyphenols, flavonoids, and tannins of the tested aqueous and organic extracts.

Ethanolic macerated had a strong inhibition against *Proteus mirabilis* (16 mm); ethanolic extract and ethanolic macerated had a bactericidal effect against *Proteus mirabilis*; these same extracts have a bactericidal effect against *Staphylococcus aureus* CECT 976 with 4 mg/ml each.

We believe and hope that this work can contribute to the improvement of traditional medicine practices and to better guide the use of this plant. In addition, the present study could open up new work perspectives, consisting on the one hand an in-depth study on the leaves of *C. humilis* by isolation, purification, and determination of the structures of the active compounds and subsequently conducting *in vivo* investigations based on the *in vitro* study of this part. On the other hand and based on the results of the ethnopharmacological survey, it would be interesting to study the pharmacological properties of the different parts of *C. humilis* used in traditional phytotherapy and also to carry out a correlation study between their chemical composition and their biological activities.

The ethnopharmacological survey is also a valuable source of data and information on the traditional use of *C. humilis* in several sectors, namely, the therapeutic and food sector for humans and animals, and also in the handicraft sector based on the dwarf palm leaves.

## Figures and Tables

**Figure 1:** 3D geographical map representing the location of the stations of the ethnopharmacological survey *on Chamaerops humilis* L. var. argentea Andre in the study area: province of Taza (north-east Morocco).

**Figure 2:** Survey stations: (a) Taza city, (b) Bab El Mrouj, (c) Gueldamane, and (d) Bab Boudir.

**Figure 3:** *Chamaerops humilis* L. var. argentea Andre (pictures taken on 16 April 2017 in Bab Boudir, located 60 km from the city of Taza; geographical coordinates: N 34°405.635′, W 004°05.900′).

**Figure 4:** Distribution of users of *C. humilis* in traditional medicine according to age group in the region of Taza, Morocco.

**Figure 5:** Medicinal uses of *C. humilis* according to gender in the region of Taza, Morocco.

**Figure 6:** Level of study of *C. humilis* users in the Taza region, Morocco.

**Figure 7:** Parts used of *C. humilis* in the region of Taza, Morocco.

**Figure 8:** Percentage of preparation methods of different parts of *C. humilis* in the region of Taza, Morocco. (a) Heart of palm; (b) spadice; (c) fruits; (d) root; (e) leaf.

**Figure 9:** Projection of individuals on the factorial plane (F1 × F2). G1: group 1; G2: group 2; G3: group 3; D: decocted; I: infused; Aq. M: aqueous macerated; EtOH: ethanolic extract; M. EtOH: ethanolic macerate; CHCL_3_: chloroformic extract; M. CHCl_3_: chloroformic macerated; Hex: hexane extract; M. Hex: hexanic macerated.

**Table 1:** Diseases treated according to the part used of *C. humilis* in the region of Taza, Morocco.

Parts of the plant *C. humilis*	Diseases treated
Palm heart	Digestive disorders, diarrhea, inflammation, diabetes, toning, cardiovascular disease, respiratory system disorders, hepatopathy
Spadice	Digestive disorders, diarrhea, inflammation, diabetes, toning, cardiovascular disease, respiratory system disorders, hepatopathy
Fruit	Digestive disorders, diarrhea, inflammation, diabetes, toning, cardiovascular disease, respiratory system disorders, hepatopathy, fertility, immune system disorders
Root	Digestive disorders, diabetes, hair loss
Leaves	Digestive disorders for humans and livestock

**Table 2:** The different uses of *C. humilis* in the region of Taza, Morocco.

Part of the plant	Type of application
Palm heart, spadice	Therapeutic
	Human alimentation

Fruit	Therapeutic
	Human alimentation
	Animal feed
	Magic

Leaves	Therapeutic
	Human alimentation
	Basketry dishwashing tool
	Magic

The entire plant	Firewood

**Table 3:** Mineral composition of *Chamaerops humilis* L. var. argentea leaves in mg/kg of plant material.

Minerals	Content in mg·kg^−1^ of dry matter
Iron (Fe)	82395.00
Potassium (K)	9354.90
Phosphorus (P)	1828.62
Magnesium (Mg)	1312.47
Sodium (Na)	627.03
Copper (Cu)	542.64
Calcium (Ca)	92.19
Zinc (Zn)	66.15
Selenium (Se)	3.00
Strontium (Sr)	3.00

**Table 4:** Yields of aqueous and organic extractions obtained from the leaves of *C. humilis*.

	Extracts	Yield in %
Aqueous extracts	**Decocted**	**10.00**
	Infused	2.20
	Aqueous macerated	1.20

Organic extracts	**Ethanolic extract**	**10.84**
	Ethanolic macerated	3.18
	Chloroformic extract	1.24
	Chloroformic macerated	1.04
	Hexanic extract	0.82
	Hexanic macerated	0.43

**Table 5:** Chemical composition of the powder and aqueous and organic extracts of the leaves of *C. humilis.*

Leaf powder/aqueous and organic extracts	Catechic tannins	Gallic tannins	Flavonoids	Saponins	Alkaloids	Sterols	Anthracenosides	Free quinones	Anthraquinones
Powder of leaves	+++	−	+	+++	−	+++	−	+	−
Decocted	+++	−	++	+++	−	−	−	+	−
Infused	+++	−	+	+	−	−	−	−	−
Aqueous macerated	+++	−	—	+++	−	−	−	−	−
Ethanolic extract	+++	−	+	++	−	−	−	++	−
Ethanolic macerated	+++	−	++	+	−		−	++	−
Chloroformic extract	+	−	−	−	−	−	−	−	−
Chloroformic macerated	++	−	−	−	−	−	−	−	−
Hexanic extract	+	−	−	−	−	++	−	−	−
Hexanic macerated	+	−	−	−	−	+++	−	−	−

(+++): strong presence; (++): medium presence; (+): weak presence; (−): absence.

**Table 6:** Total polyphenol, flavonoid, and catechic tannin contents of aqueous and organic extracts of *C. humilis* leaves.

	Extracts	Total polyphenols (*μ*g GAE/mg E)	Flavonoids (*μ*g QE/mg E)	Catechic tannins (*μ*g CE/mg E)
Aqueous extracts	Decocted	13.23 ± 0.19^a^	56.36 ± 0.39^a^	10.08 ± 0.07^a^
	Infused	2.11 ± 0.03^b^	41.94 ± 0.09^a^	1.28 ± 0.03^a^
	Aqueous macerated	2.02 ± 0.04^b^	4.48 ± 0.26^a^	1.26 ± 0.04^a^

Organic extracts	Ethanolic extract	96.99 ± 0.82^c^	457.98 ± 5.18^b^	50.27 ± 0.99^b^
	Ethanolic macerated	100.27 ± 0.66^c^	468.25 ± 9.07^b^	52.11 ± 0.24^b^
	Chloroformic extract	28.04 ± 0.43^d^	356.87 ± 10.90^c^	35.72 ± 2.35^c,d^
	Chloroformic macerated	37.51 ± 1.66^e^	542.70 ± 24.03^d^	39.05 ± 0.78^d^
	Hexane extract	20.80 ± 1.33^f^	273.25 ± 8.92^e^	25.50 ± 0.51^e^
	Hexanic macerated	34.77 ± 1.19^e^	335.48 ± 10.67^c,e^	30.16 ± 1.02^c,e^

All results presented are the mean of three individual replicates ( = 3 ± SEM). Values with the same superscript letters in the same row are not significantly different (*p* < 0.05).

**Table 7:** Antioxidant activity of aqueous and organic extracts of *C. humilis* leaves.

Extracts/tests		H_2_O_2_ (%)	DPPH (IC_50_) (*μ*g/ml)	ABTS (mg TE/g E)	FRAP (mg TE/g E)	RP (mg AAE/g E)
Aqueous extracts	Decocted	45.77 ± 0.15^a^	6814.00 ± 0.08^a^	14.44 ± 0.003^a^	23.44 ± 0.07^a^	2.46 ± 0.04^a^
	Infused	29.65 ± 0.31^b^	10280.00 ± 0.04^a^	2.49 ± 0.19^a^	6.67 ± 0.017^b^	2.49 ± 0.01^a^
	Aqueous macerated	29.24 ± 0.62^b^	9260.00 ± 0.39^a^	2.46 ± 0.05^a^	5.34 ± 0.14^c^	0.31 ± 0.007^a^

Organic extracts	Ethanolic extract	36.80 ± 0.33^c^	44.25 ± 2.31^a^	78.21 ± 0.98^b^	144.71 ± 0.35^d^	10.14 ± 0.04^b^
	Ethanolic macerated	37.34 ± 0.55^d,c^	31.18 ± 0.66^b^	108.28 ± 1.29^c^	148.85 ± 0.43^e^	10.86 ± 0.01^c^
	Chloroformic extract	34.83 ± 0.26^e,c^	490.06 ± 0.54^c^	30.10 ± 0.75^d^	16.77 ± 0.69^f^	1.14 ± 0.05^d^
	Chloroformic macerated	35.79 ± 0.29^f,c,d,e^	491.53 ± 2, 08^d,b,c^	41.93 ± 0.62^e^	17.21 ± 0.10^g,f^	2.12 ± 0.05^e^
	Hexanic extract	33.96 ± 0.17^g,e,f^	975.83 ± 11.83^e,b,c,d^	14.87 ± 2.31^f^	9.53 ± 0.23^h^	0.92 ± 0.07^f,d^
	Hexanic macerated	21.59 ± 1.14^h^	335.10 ± 0.5^f,d,e^	30.15 ± 3.76^g,d^	39.62 ± 0.08^i^	1.41 ± 0.02^g^

Reference standards	Ascorbic acid	14.35 ± 0.002^i^	0.17 ± 0.02^g,b,c,d,e,f^	—	—	—
	BHT	—	1.59 ± 0.13^h^	—	—	—
	Trolox	—	1.75 ± 0.09^i^	—	—	—

All results expressed are the mean of three individual replicates ( = 3 ± SEM). Values with the same superscript letters in the same row are not significantly different (*p* < 0.05).

**Table 8:** Antibacterial activity of organic extracts from the leaves of *C. humilis.*

Extracts/bacterial strains	Ethanolic extract (mg/ml)			Ethanolic macerated (mg/ml)			Chloroformic extract (mg/ml)			Chloroformic macerated (mg/ml)			Hexanic extract (mg/ml)			Hexanic macerated (mg/ml)			Standard (−) (*μ*g/ml)	Standard (+)
	**40**	**80**	**100**	**40**	**80**	**100**	**40**	**80**	**100**	**40**	**80**	**100**	**40**	**80**	**100**	**40**	**80**	**100**	**T/AK 20/30**	**DMSO (10%)**
	Inhibition zone (mm)																			
*E. coli*	—	7	8	—	7	8	—	7	8	—	—	—	—	—	—	—	7	7	12/T	—
*P. m*	7	**12**	**12**	11.5	**16**	**16**	7	9	10	—	—	—	—	—	—	8	9	9	22/T	—
*P. a*	—	7	8	—	7	8	—	7	8	—	—	—	—	—	—	—	7	8	27/AK	—
*S. a*	—	7	8	—	7	8	—	7	8	—	—	—	—	—	—	—	7	8	12/T	—
*Lis*	—	7	8.5	9	**14**	**14**	—	7	8	—	—	—	—	—	—	—	7	9	11/T	—
*B. s*	—	7	8	10.5	10	**14**	—	7	7.5	—	—	—	—	—	—	7	7	8	10/T	—

T: tetracycline; AK: amikacin; *E. coli*: *Escherichia coli*; *P. m*: *Proteus mirabilis*; *P. a*: *Pseudomonas aeruginosa* CECT 118; *S. a*: *Staphylococcus aureus* CECT 976; *B. s*: *Bacillus subtilis* DSM 6633; *Lis*: *Listeria innocua* CECT 4030; (−): absence of inhibition.

**Table 9:** Minimum inhibitory concentration (MIC) and minimum bactericidal concentration (MBC) of organic extracts from the leaves of *C. humilis*.

Extracts/bacterial strains	Ethanolic extract			Ethanolic macerated			Chloroformic extract			Hexanic macerated		
	MIC	MBC	MBC/MIC	MIC	MBC	MBC/MIC	MIC	MBC	MBC/MIC	MIC	MBC	MBC/MIC
	mg/ml			mg/ml			mg/ml			mg/ml		
*E. coli*	*5*	ND	—	*2.5*	80	32	20	80	*4*	10	ND	—
*P. m*	20	40	**2**	10	40	*4*	10	80	8	10	40	*4*
*P. a*	10	40	*4*	*2.5*	40	16	10	80	8	5	ND	—
*S. a*	20	80	*4*	10	40	*4*	40	80	**2**	20	ND	—
*Lis*	*5*	80	16	*2.5*	40	16	*1.25*	40	32	*2.5*	80	32
*B. s*	40	ND	—	5	ND	—	5	ND	—	20	ND	—

*E. coli*: *Escherichia coli*; *P. m*: *Proteus mirabilis*; *P. a*: *Pseudomonas aeruginosa* CECT 118; *S. a*: *Staphylococcus aureus* CECT 976; *B. s*: *Bacillus subtilis* DSM 6633; *Lis*: *Listeria innocua* CECT 4030; MBC/MIC ≤ 4: bactericidal power; MBC/MIC > 4: bacteriostatic power; ND: not determined.

**Table 10:** Correlation matrix between phytochemical data (total polyphenols, flavonoids, and catechic tannin contents) and antioxidant activity via the five tests (H_2_O_2_, DPPH, ABTS, FRAP, and RP) of *C. humilis* leaves.

Variables	H_2_O_2_	DPPH	ABTS	FRAP	RP	Total polyphenols	Flavonoids	Catechic tannins
H_2_O_2_	**1**							
DPPH	0.0543	**1**						
ABTS	0.2503	**0.9214**	**1**					
FRAP	0.2240	0.8377	**0.9341**	**1**				
RP	0.3280	0.7581	**0.9104**	**0.9743**	**1**			
Total polyphenols	0.2142	**0.9418**	**0.9779**	**0.9644**	**0.9271**	**1**		
Flavonoids	0.0676	**0.8897**	0.7599	0.5584	0.4982	0.7559	**1**	
Catechic tannins	0.1619	**0.9753**	**0.8843**	0.7472	0.6812	**0.8924**	**0.9532**	**1**

## Data Availability

The survey data was collected using an anonymous questionnaire; the datasets used and analyzed are included in the article in the form of tables and figures.

## Abbreviations

ICP-AES: Inductively coupled plasma atomic emission spectrometry
*C. humilis*: *Chamaerops humilis* L. var. argentea Andre
Fe: Iron
K: Potassium
P: Phosphorus
Mg: Magnesium
Na: Sodium
Cu: Copper
Ca: Calcium
Zn: Zinc
Se: Selenium
Sr: Strontium
AlCl_3_: Aluminum chloride
GAE: Gallic acid equivalent
QE: Quercetin equivalent
CE: Catechin equivalent
H_2_O_2_: Hydrogen peroxide
DPPH: 1,1-Diphenyl-2-picrylhydrazyl
ABTS: 2,2-Azino-bis-3-ethylbenzothiazolin-6-sulfonic acid
FRAP: Ferric-reducing ability of plasma
RP: Iron-reducing power
TE: Trolox equivalent
AAE: Ascorbic acid equivalent
BHT: Butylated hydroxytoluene
ANOVA: Analysis of variance
PCA: Principal component analysis
GA: Gallic acid
Q: Quercetin
IC_50_: Concentration that causes 50% inhibition
DMSO: Dimethyl sulfoxide
CFU: Colony-forming unit
T: Tetracycline
AK: Amikacin
*E. coli*: *Escherichia coli*
*Pm*: *Proteus mirabilis*
*Pa*: *Pseudomonas aeruginosa* CECT 118
*Sa*: *Staphylococcus aureus* CECT 976
*Bs*: *Bacillus subtilis* DSM 6633
*Lis*: *Listeria innocua* CECT 4030
MTT: 3-(4,5-Dimethylthiazol-2-yl)-2,5-diphenyl tetrazolium bromide
MIC: Inhibitory concentrations
MBC: Minimum bactericidal concentrations.
